RETRACTED

# Analysis of the Effect of Branched Chain Amino Acids on Muscle Health Information of Swimmers Based on Multisensor Fusion and Deep Learning

**DOI:** 10.1155/2022/2573058

**Published:** 2022-04-26

**Authors:** Shimeng Huang, Qiulan Luo, Jingwen Liao

**Affiliations:** ^1^Swimming Teaching and Research Office, Guangzhou Sport University, Guangzhou, 510500 Guangdong, China; ^2^Department of Sports, Central China Normal University, Wuhan, 430070 Hubei, China; ^3^Science Experiment Center, Guangzhou Sport University, Guangzhou, 510500 Guangdong, China

## Abstract

Swimmers must fully mobilize the muscles of the whole body during exercise, and it is necessary to study the protection of swimmers from muscle damage. Now, muscle damage is increasing year by year, and more athletes are affected. Therefore, studying the causes of muscle injuries and exploring more effective treatments have become important research topics in the field of sports medicine. This study is mainly based on deep learning to analyze the protective effect of branched-chain amino acids on swimming athletes' muscle injury. Due to the complex and changeable environment and the interference of unknown factors, a single sensor cannot meet the needs of obtaining information. Therefore, people have developed the technology of multisensor information fusion to obtain enough information. Multisensor data fusion technology can synthesize the information of each sensor and then obtain more comprehensive and accurate decision-making information. This study is mainly based on multisensor fusion and deep learning to analyze the impact of branched chain amino acids on Swimmers' muscle health information. Finally, two experiments were designed in this article. The first experimental result showed that the pain level of the experimental group who took BCAA supplements was 19% lower than that of the control group that did not take the BCAA supplement within three days after exercise. The results of the second experiment show the following: after exercise, the creatine kinase activity value of the experimental group taking BCAA supplement was 4.38 ± 1.45, and the creatine kinase activity value of the control group taking placebo was 5.42 ± 2.12. It proves that BBCA can protect muscle damage by reducing the activity of creatine kinase.

## 1. Introduction

### 1.1. Background

Muscle health is an essential information for athletes. Once muscle injury occurs, it will break the ring of muscle health. The cause of muscle damage is overload and repeated exercise. For example, some are hereditary, some are drug-induced, hereditary muscle damage is muscular dystrophy, and it may be caused by some strains, impacts, or bacterial infections, which can also easily cause some muscle damage. Scientific training methods and moderate stimulation can effectively promote the increase of the transverse area of skeletal tendons, thereby increasing muscle strength. Wrong methods and overloaded exercise may easily cause muscle pain, swelling, decreased contractility, and muscle damage. There are various injury methods and different degrees of muscle injury, and clinical research is more difficult. The protein content of branched chain amino acids is high. For athletes, supplementing branched chain amino acids can greatly relieve fatigue and improve their sports ability. In this context, we analyze the effect of branched chain amino acids on muscle health information of swimmers.

RETRACTED

### 1.2. Significance

Muscle health is an important guarantee for swimmers' physical quality and skill level. However, muscle injury is a common sport injury of swimmers. Once muscle injury is caused, it may be a continuous injury for swimmers. After muscle strain and severe pain at the strained site, cord-like lumps formed by muscle tension can be felt on hands, obvious pain on the touch, local swelling or subcutaneous hemorrhage, and significantly restricted activity. Many studies have shown that the supplement of branched-chain amino acids during exercise can effectively promote protein assimilation during the recovery period after exercise. It accelerates muscle protein synthesis, prevents the deterioration of muscle tissue, reduces exercise-induced muscle damage, and prolonged muscle soreness.

### 1.3. Related Work

Branched-chain amino acids are important essential amino acids for the human body and participate in various physiological activities of the human body. Therefore far, many scholars have studied it, trying to analyze its function in the human body. Sun et al. performed transcriptomics and metabolomics analysis on the failing hearts of mice caused by pressure overload. They found that inhibition of gene expression of branched-chain amino acid catabolism was confirmed to exist in the heart of human cardiomyopathy. Sun et al.'s research using genetic mouse models has shown that branch-chain amino acid catabolism defects promote heart failure and are related to oxidative stress and metabolic disorders caused by mechanical load. However, their experimental data are less [1]. Duan et al. studied the effects of BCAA ratio on intramuscular fat content and fatty acid composition in different parts of growing pigs and detected the mRNA expression level of lipid metabolism-related genes in these muscle tissues. The results show that the low egg diet with BCAA ratio in the range of 1 : 0.25 : 0.25–1 : 0.75 : 0.75 can maximize the IMF content in muscle, which is a complex test method [2]. Kikuchi et al. randomly divided patients undergoing major hepatocellular carcinoma surgery into two groups. One group started taking BCAA 3 weeks before liver resection, and the other group was a non-BCAA group. BCAA has a significant effect on preventing ascites and pleural effusion and improving albumin metabolism. However, there are too many experimental factors [3]. The metabolism of BCAA in Trypanosoma cruzi mainly depends on its transport into the cell. In this work, Manchola et al. described the BCAA transport of Trypanosoma cruzi using a kinetic method. Their data indicate that BCAA is transported by a single saturated transport system that can recognize leucine, isoleucine, and valine. However, his content is not new enough [4]. Connelly et al. studied the relationship between changes in leptin and adiponectin levels in individuals with different degrees of glucose tolerance and the degree of association between BCAA and insulin resistance. BCAA is related to insulin resistance. After adjusting for age, gender, T2DM, BMI, and leptin and adiponectin, this correlation still exists. The study lacks more comparative design [5].

RETRACTED

### 1.4. Innovation

The innovation of this article is (1) combining deep learning with branched-chain amino acids; this paper describes the function prediction method of branched-chain amino acids based on deep learning, which is innovative in this method. (2) The design experiment proved that branched chain amino acids have the function of reducing delayed soreness and injury protection to muscles, and it is innovative in experiments.

## 2. Muscle Injury Protection Method Based on Deep Learning

### 2.1. Deep Learning

Deep learning is a machine learning algorithm, which is currently very useful for the interpretation of text, image, and sound data. The concept of deep learning comes from the study of artificial neural networks. Compared with shallow artificial neural networks, “depth” is a significant feature of deep learning. It can be understood as a deep neural network, and its model is characterized by multiple hidden layers. Layer perceptron: the effect of deep learning on sound and image recognition is in a leading position, surpassing traditional algorithms. There are many representative algorithms for deep learning [6, 7]; here are a few introductions.

1. Convolutional neural network

In 1962, Hubel et al. were inspired by cell biology and proposed a convolutional neural network with reference to the arrangement of visual cell tissue. Convolutional neural networks are constructed by imitating the visual perception mechanism of biology and can perform supervised learning and unsupervised learning and small computational effort to learn grid-like topology features, such as pixels and audio, with stable effects and no additional feature engineering requirements on the data. The convolutional neural network mainly contains a 3-layer structure. It first inputs the picture into the network through the input layer, the convolutional layer, and the pooling layer together form the second layer to process the picture. Its structure is shown in Figure 1.

RETRACTED

Activation functions have been widely used in many neural networks, and different types of activation functions have completely different effects. The result of the sigmoid function is a constant positive value distributed between 0 and 1. When the size of *x* gradually approaches infinitesimal or infinite, its gradient value gradually approaches 0, which leads to the phenomenon of gradient dispersion. The curve of the sigmoid function presents a monotonous increasing trend, which is easy to optimize. As a result, the weights of the neural network can only be updated in one direction, and the convergence speed is slow [8]. The formula of the sigmoid function is:

(1) $$\begin{array}{c} \text{Sigmoid}\left(x\right)=\frac{1}{1+e^{-x}}. \end{array}$$

The Tanh function is also called the hyperbolic tangent function. Its output is a value between -1 and 1, and the expected value is 0. When the size of *x* gradually approaches positive infinity or negative infinity, its gradient value gradually approaches 0. Therefore, the Tanh function is essentially a modification of the sigmoid function, which inherits the advantages of the sigmoid function [9]. However, it still has not solved a series of problems that plague convolutional neural networks. The formula of the Tanh function is as follows:

(2) $$\begin{array}{c} \text{Tanh}\left(x\right)=\frac{e^{x}-e^{-x}}{e^{x}+e^{-x}}. \end{array}$$

The ReLU function has a strong mathematical and biological foundation. The ReLU function sets the value of the negative value interval of *x* to 0, and the value of the positive value interval does not change. When the input is a negative number, the neural node will not produce a response operation. It means that at the same time, only a part of the neural nodes produce a response. This working mechanism causes the neurons of the neural network to have the characteristics of sparse activation, which greatly improves the calculation speed. Compared with the first two activation functions, since the ReLU function does not have a saturation zone, there is no series of problems that plague the first two activation functions during the training process. Therefore, the application range of the ReLU function is wider [10]. The formula is as follows:

(3) $$\begin{array}{c} f\left(x\right)=\max\left(0,x\right). \end{array}$$

Figure 2 shows the images of the three functions.

RETRACTED

Convolutional neural networks are inspired by the working mechanism of biological systems. Neural nodes do not need to perceive all visual information, but only need to be sensitive to visual locally associated information. The correlation information between the deep spatial and local features in the convolutional neural network is integrated into the global correlation information. Therefore, the unique design mode and working mechanism of convolutional neural network make it have strong applicability. Without a large number of parameters and neural nodes, it effectively extracts the spatial characteristics of the input information, which greatly reduces the risk of overfitting.

(2) Recurrent neural network

Recurrent neural networks are mainly used to process a series of data sequences arranged in a specific time sequence. In traditional neural networks, neurons in different layers are combined with each other in a fully connected manner. However, the neurons in each layer are not connected to each other, and they are powerless to process information that has a logical relationship between the front and back [11]. For example, to infer the next sentence from one sentence, it needs to know the content of the previous sentence, because the content of the next sentence is the result of inference based on the previous sentence. In short, the cyclic neural network not only processes the characteristics of the current input information but also processes the logical relationship of the input information. When a sequence of data is input to the cyclic neural network, the cyclic neural network first stores the previous input data. When the subsequent sequence information is input, the state information stored in the front is called to participate in the calculation of the output result. In the cyclic neural network, each node is connected to each other, and the previous output results jointly participate in the processing of the current state sequence information. The general process of cyclic neural network is shown in Figure 3.

The forward propagation algorithm of the recurrent neural network is:

(4) $$\begin{array}{c} h_{t}=\sigma \left(Ax^{t}+Bh^{t-1}+p\right), \end{array}$$

(5) $$\begin{array}{c} Q_{t}=Ch_{t}+c, \end{array}$$

(6) $$\begin{array}{c} y_{t}^{,}=\text{softmax}\left(Q_{t}\right). \end{array}$$

Among them, *h*_*t*_ represents the state of the hidden layer, *Q*_*t*_ is the output result at time *t*, and *y* is the actual output result of the model at time *t*. *A*, *B*, and *C* are the linear parameters of the recurrent neural network [12], *σ* represents the activation function, and *p* is the bias function.

RETRACTED

The calculation parameters are continuously updated through gradient descent, and the final *A*, *B*, *C*, and other parameters of the recurrent neural network model are obtained. The gradient calculation formula of parameter *C* is as follows:

(7) $$\begin{array}{c} \frac{\partial L}{\partial C}=\overset{\tau }{\underset{t=1}{\sum }}\frac{\partial L_{t}}{\partial C}=\overset{\tau }{\underset{t=1}{\sum }}\left(y_{t}^{,}-y_{t}\right)∙h_{t}^{T}. \end{array}$$

The gradient loss at a certain moment is determined by the gradient at the present moment and the loss value at the next moment. The formula is as follows:

(8) $$\begin{array}{c} \sigma_{t}=\frac{\partial L}{\partial h_{t}}, \end{array}$$

(9) $$\begin{array}{c} \sigma_{t}=\left(y_{t}^{,}-y_{t}\right)∙C^{T}+B^{T}∙\sigma^{t+1}\mathrm{diag}\left(1-{\left(h^{t+1}\right)}^{2}\right). \end{array}$$

The numerical value in formula (8) can be enlarged or reduced proportionally. The calculation expressions of parameters *A*, *B*, and *p* are:

(10) $$\begin{array}{c} \frac{\partial L}{\partial B}=\overset{\tau }{\underset{t=1}{\sum }}\mathrm{diag}\left(1-{\left(h^{t}\right)}^{2}\right)∙\sigma^{t}∙{\left(h^{t-1}\right)}^{T}, \end{array}$$

(11) $$\begin{array}{c} \frac{\partial L}{\partial p}=\overset{\tau }{\underset{t=1}{\sum }}\mathrm{diag}\left(1-{\left(h^{t}\right)}^{2}\right)∙\sigma^{t}, \end{array}$$

(12) $$\begin{array}{c} \frac{\partial L}{\partial A}=\overset{\tau }{\underset{t=1}{\sum }}\mathrm{diag}\left(1-{\left(h^{t}\right)}^{2}\right)∙\sigma^{t}∙{\left(x^{t}\right)}^{T}. \end{array}$$

From a theoretical analysis, the recurrent neural network can handle serialized data very well. However, when applied to the actual production environment, its application effect is often troubled by problems such as gradient disappearance [13].  Figure 4 is a schematic diagram of the structure of a long- and short-term neural network.

There are four network layers in the chain structure module. The long- and short-term memory network deletes or adds changes to the characteristic information in the network through a gate control structure, and the gate can selectively modify the characteristic information. The gate control mainly uses the sigmoid layer and a dot multiplication operation to filter and combine information. There are three gates in a single unit of the entire long- and short-term memory network to control the selection or storage state of the input feature information. We call them feature information input gates, feature information output gates, and feature information forget gates [14].

RETRACTED

### 2.2. Functional Prediction of Branched Chain Amino Acids in View of Deep Learning

1. Overview of branched chain amino acids

Branched-chain amino acids are an important energy sources. Oxidative decarboxylation generates ATP for energy. BCAA is an essential amino acid and an indispensable nutrient for the human body [15]. They can only be obtained from the external food they ingest, and they are not synthesized or synthesized in a small amount in the body. As one of the branched chain amino acids, leucine occupies a large proportion of the amino acids that make up the protein, and it is the main product of protein catabolism. BCAA is a large molecule neutral amino acid. The classification diagram is shown in Figure 5.

(2) Functional evaluation and measurement of branched chain amino acids

The function prediction problem of branched-chain amino acids can be converted into a multilabel learning problem for research, so its evaluation indicators use common indicators in multilabel learning [16]. First of all, we should understand the value of *F*1. *F*1 is calculated based on the accuracy rate (precision) and recall rate (recall); the formula is as follows:

(13) $$\begin{array}{c} P=\frac{\text{BP}}{\text{BP}+\text{FP}}, \end{array}$$

(14) $$\begin{array}{c} R=\frac{\text{BP}}{\text{BP}+\text{FN}}, \end{array}$$

(15) $$\begin{array}{c} \text{Presion}=\frac{\sum_{i=1}^{N}P}{N}, \end{array}$$

(16) $$\begin{array}{c} \text{Recall}=\frac{\sum_{i=1}^{N}R}{N}, \end{array}$$

(17) $$\begin{array}{c} F1=\frac{\sum_{i=1}^{N}\left(\left(2PR/P\right)+R\right)}{N}. \end{array}$$

In the formula, *B* is the true functional marker of amino acids, the functional predictive value of branched-chain amino acids is *P*, TP, and FP are the number of true positive and false positives, respectively, and FN is the number of false negatives. *P* represents the accuracy rate, and *R* represents the recall rate.

(3) The prediction process of branched-chain amino acids based on deep learning

- Use LSTM to extract sequence long-range information

This chapter uses a three-layer two-way long- and short-term memory network to mine the long-range feature information in the branched-chain amino acid sequence. The long- and short-term memory network is proposed to solve the gradient explosion problem in the network. The long- and short-term memory networks have one more gate unit mechanism than traditional recurrent neural networks. The gate unit mechanism determines the information selection and storage and dissemination of the entire long- and short-term memory network module [17]. Here, a three-layer two-way long- and short-term memory network is used to extract the feature information of the interaction between the branched-chain amino acid sequences, and the fusion feature *f*_*n*_ in two directions is obtained.

(18) $$\begin{array}{c} f_{n1}=\text{LSTM}\left(f_{n1}^{s-1},f_{n1-1}^{s}\right), \end{array}$$

(19) $$\begin{array}{c} f_{n2}=\text{LSTM}\left(f_{n2}^{s-1},f_{n2-1}^{s}\right), \end{array}$$

(20) $$\begin{array}{c} f_{n}=f_{n1}⊕f_{n2}. \end{array}$$

*f*_*n*1_ and *f*_*n*2_ represent the forward and reverse feature information representation of the *t*th position, and ⊕ represents the fusion of the forward and reverse feature information.

(ii) Predictive classification

The classification layer of this module completes the final prediction. The input layer accepts the feature vector combined with the three-layer two-way LSTM, and the hidden layer uses the activation function ReLU function to perform the output activation operation [18]. The output layer uses the Softmax function, which calculates and predicts the size of each probability distribution:

(21) $$\begin{array}{c} p_{t}=\text{softmax}\left[\text{relu}\left(W_{i}f+c_{i}\right)\right], \end{array}$$

(22) $$\begin{array}{c} \text{softmax}\left(z\right)=\frac{e^{z}}{\sum e^{z}}. \end{array}$$

In the formula, *W*_*i*_ represents the weight of the *i*th layer in the network layer, and *c*_*i*_ represents the bias of the *i*th layer in the network layer. *p*_*t*_ is the predicted probability of the *t*th branched chain amino acid in the amino acid sequence.

RETRACTED

### 2.3. Muscle Protection Methods Based on Branched Chain Amino Acids

The impact of muscle injury on athletes is enormous. At present, researches on sports injuries are attached great importance at home and abroad. A series of research results ensure the physical and mental health of athletes and provide a lot of motivation for the sustainable development of various sports [19].

1. Muscle damage

Muscle damage is widespread in sports, mainly due to local muscle overload or repeated exercise. It may be clinically manifested as various degrees of pain and dysfunction. The treatment of muscle injury mainly includes preservation treatment and surgical treatment such as ice compression, hemostasis, analgesia, and fixation. At present, the types of muscle injury mechanisms are shown in Figure 6.

Moreover, in sports training, preventing muscle damage is also essential. If proper warm-up exercises and stretching exercises are performed before formal training and exercise, the temperature of the muscles will rise and the mobility of the joints will increase. The viscosity of the muscle decreases, and the contraction of the muscle becomes larger, which can reduce the damage of the muscle.

(2) Steps to prevent muscle damage

The muscle injury prevention research program is divided into 4 steps, as shown in Figure 7. First, the scope of injury should be established based on the incidence and severity of muscle injury. Coaches must continuously monitor the risk factors of athletes' sports injuries during training and competitions. The second step is to determine the risk factors and injury mechanism and analyze the cause of the injury. The third step is to summarize the methods that may reduce the risk of injury and reduce the severity of injury based on the information about the risk factors and injury mechanism. Finally, the first step must be repeated to evaluate the effectiveness of these methods.

(3) Protection of branched chain amino acids on muscles

High-intensity exercise training may cause chronic muscle pain or changes in the activity of certain serum enzymes. BCAA protects the structure and function of the muscle cell membrane. It prevents the overflow and release of intracellular enzymes, inhibits lipid peroxidation, and reduces calcium overload. It uses mitochondrial energy to maintain and prevent membrane structure and function, and protect muscles from damage. Delayed muscle soreness usually occurs after a certain period of inappropriate high-intensity exercise, and BCAA can reduce this pain. The role of BCAAs in scavenging free radicals and maintaining the normal function of cell membranes has a positive effect on the weakening the impact of DOMS.

RETRACTED

## 3. Branched Chain Amino Acids' Muscle Protection Experiments on Swimming Athletes

### 3.1. The Effect of Branched Chain Amino Acids on Delayed-Onset Muscle Soreness

The causes of delayed muscle soreness have been explained above.

1. Research object

Selecting juniors majoring in swimming from a sports college, 40 men and women each aged between 18 and 22. Their physical parameters are shown in Table 1. The selected athletes have similar body types and exercise levels. These athletes averaged more than 3 exercises per week and stopped strenuous exercise three days before the experiment. This experiment also tests their physical fitness to ensure that their physical conditions are suitable for this experiment.

(2) Experimental process

The athletes were divided into an experimental group and control group. There are 40 people in each group, and 20 people in each male and female groups. The grouping follows the principle of randomization. During the experiment, we first use the numerical rating scale to evaluate the pain level of all athletes. After the assessment, each athlete was allowed to swim 100 meters for a total of 5 times, and the pain level test was performed immediately after the swim. After the test, the experimental group took BCAA supplements. For the next 72 hours, the experimental group was given branched chain amino acid (BCAA) supplements every 24 hours, and the control group did not take any drugs. And during these 72 hours, the athletes were tested for pain levels every 12 hours.

(3) Pain grade evaluation

The numerical rating scale is used to measure the magnitude or intensity of pain. It uses 11 numbers from 0 to 10. This experiment uses a numerical rating scale to grade athletes' muscle pain. The higher the level, the higher the degree of pain. The numerical rating scale has high reliability and is suitable for this experiment.

(4) The choice of BCAA supplements

The BCAA product selected in this experiment is Scivation Xtend supplement. Its ingredients include 7000 mg of branched chain amino acids (2 : 1 : 1). In terms of ingredients, this product has reached a relatively high amino acid drink specification. The main function of Scivation Xtend is to provide fuel for muscles, maintain muscle anabolism, and maintain fluid balance. Its branched chain amino acids are quickly absorbed.

(5) Experimental results and analysis

We conducted a three-day pain rating for the athletes and averaged the pain levels of the two groups of athletes. The results of the athletes' pain ratings obtained are shown in Figure 8.

RETRACTED

The maximum pain level of the experimental group that took the BCAA supplement group appeared just after the exercise, with a value of 2.2. In the subsequent pain rating, the pain level of the experimental group gradually decreased. In the control group, the maximum pain level of the group that did not take any drugs was 2.5 at 24 hours after exercise. The pain level of this group gradually increased before 24 h after exercise. After 24 hours, the pain level gradually decreased. By calculation, within three days after exercise, the pain level of the experimental group was reduced by 19% compared with the control group. It can be concluded that the reason for the gradual decrease in the pain level of the experimental group after exercise is the use of BCAA supplements. It can prove that BCAA has a certain relieving effect on delayed-onset muscle soreness, and it reduces the athlete's pain level by 19% within three days after exercise.

In addition to the statistical results and evaluation of all athletes, this experiment also tried to study whether gender differences affect the effect of BCAA. Separating male and female statistics of the average pain level, the results are shown in Figure 9.

For male athletes, there is little difference in pain levels between the experimental group and the control group, respectively, 2.3 and 2.3. The highest pain levels in both groups appeared just after exercise. Between 12 h and 72 h after the exercise, the average pain level of male athletes decreased. However, the pain level of the experimental group that took the BCAA supplement group was always slightly lower than that of the control group. It proves that BCAA can still relieve delayed soreness in male athletes, but the effect is not obvious. For female athletes, the maximum pain level of the experimental group appeared just after exercise. The control group appeared 24 h after exercise, and between 12 h and 72 h after exercise. The average pain level of the experimental group was significantly lower than that of the control group. It can be seen that BCAA supplements are more effective in reducing delayed muscle soreness for female athletes.

RETRACTED

### 3.2. Protective Experiment of Branched Chain Amino Acids on Muscle Injury

1. Research object

The subjects of this experiment are 30 swimmers from a district-level swimming team. All athletes are in good physical condition, have no medical history that affects the experiment, and have not taken any drugs or nutrients related to increased muscle strength in the past month. And their height and body shape are similar, and their physical parameters are shown in Table 2. Before the experiment, inform the experiment process and experiment purpose, and the subjects will participate voluntarily. The 30 athletes were divided into two groups, the experimental group and the control group.

(2) Experimental process

Athletes shall not perform high-intensity exercise within 48 hours before the test, and they shall be fully warmed up under the guidance of a professional physical coach before the test. From the day the test started, the experimental group took BCAA supplements every day. The control group took a placebo every day, and the placebo was designed as a starch supplement that was similar in appearance and taste to the BCAA supplement. The test time is two weeks. During these two weeks, all swimmers have undergone normal swimming training.

After all athletes have taken BCAA supplements or placebo as required to train for two weeks, the formal test will begin. Before the test, blood samples were collected from all athletes, after which all athletes completed the 1000 m freestyle at their fastest speed, collecting blood samples again after swimming, taking blood samples 30 minutes after swimming, and measuring the activity values of glutamate (ALT) and creatine kinase (CK) in the samples.

(3) Statistical methods

The statistical analysis of CK was carried out using SPSS, and the data before and after the experiment and between the groups were analyzed for significant differences, and the significance level *P* was set to 0.05. After the activity value of ALT is counted, the average value of the activity value is taken.

(4) Experimental results

The average value of the ALT activity of glutamic acid in the three blood tests of the experimental group and the control group was calculated, and the results are shown in Figure 10.

RETRACTED

The results showed that there was no significant difference in alanine aminotransferase values between the two groups before, after, and 30 minutes after exercise, indicating that BCAA had no significant effect on the content of alt.

Counting the activity values of creatine kinase (CK) in the three blood tests of the experimental group and the control group, the results obtained are shown in Table 3.

There was no significant difference in CK content between the two groups before exercise. However, after the exercise, the difference is obvious. The CK activity value of the experimental group was significantly lower than that of the control group after exercise and 30 minutes after exercise. The intensity of exercise load is one of the main reasons for the increase in serum enzyme activity, which can also be known from the table. For the two groups, the creatine kinase activity after exercise was significantly higher than that before exercise, while the increase in the experimental group was less than that in the control group, which proved that BCAA had a significant protective effect on muscle injury.

## 4. Discussion

Having a healthy physique is the basis for athletes to train and compete, especially the muscle health information is essential for the level of swimmers, but muscle injuries often occur in swimmers. Competitive swimming is the second largest event in the Olympic Games. Therefore, it is essential to study how to protect athletes from muscle injury. Supplementing exogenous branched chain amino acids can reduce the increase in serum enzyme activity caused by exercise and protect the muscles from damage. And it can reduce muscle delayed neck soreness, which is of great significance to muscle damage. For some of the content you said is a little different from the above content, I have deleted the corresponding content.

## 5. Conclusion

This article designs experiments to verify that branched-chain amino acids can not only reduce delayed-onset muscle soreness but also protect muscle damage by reducing the activity of creatine kinase after exercise. The specific experimental results are as follows: (1) within three days after exercise, the pain level of the experimental group who took the BCAA supplement was reduced by 19% compared with the control group who did not take the BCAA supplement. (2) After exercise, the creatine kinase activity value of the experimental group taking BCAA supplement was 4.38 ± 1.45, and the creatine kinase activity value of the control group taking placebo was 5.42 ± 2.12. It proves that BBCA protects muscle damage by reducing the activity of creatine kinase. Almost all branched-chain amino acids are metabolized in skeletal muscle and play a major role in the regulation of muscle mass, while other essential amino acids are metabolized in the liver. In the near future, information research based on multisensor fusion and deep learning will be further developed.

RETRACTED

## Figures and Tables

**Figure 1:** Schematic diagram of convolutional neural network structure.

**Figure 2:** Three function images.

**Figure 3:** Recurrent neural network.

**Figure 4:** Long-short-term memory network.

**Figure 5:** Classification of branched chain amino acids.

**Figure 6:** Classification of muscle injury mechanisms.

**Figure 7:** Steps to prevent muscle damage.

**Figure 8:** Athlete's degree of pain.

**Figure 9:** Pain levels of male and female athletes.

**Figure 10:** ALT values of the two groups at different times.

**Table 1:** Basic situation of athletes.

	Age	Height	Weight	BMI
Boy	20 ± 2	172.2 ± 3.5	66.1 ± 7.1	22.6 ± 3.7
Girl	20 ± 2	160.12 ± 2.8	58.6 ± 9.2	23.5 ± 4.2
Average	20 ± 2	166.16 ± 18.15	62.25 ± 8.15	23.05 ± 3.95

**Table 2:** Basic situation of research objects.

Index	Numerical value
Age	21.1 ± 3.56
Height	175.3 ± 6.23
Weight	70.2 ± 8.68
Training years	4.22 ± 3.19

**Table 3:** Creatine kinase activity value.

	Before exercise	After exercise	30 min after exercise
Experience group *N* = 15	3.88 ± 1.12	4.38 ± 1.45	4.58 ± 1.95
Control group *N* = 15	3.86 ± 0.93	5.42 ± 2.12	5.79 ± 1.76
Difference	No	Yes	Yes

## Data Availability

Data sharing is not applicable to this article as no datasets were generated or analysed during the current study.
